# The Integrative Effects of Cognitive Reappraisal on Negative Affect: Associated Changes in Secretory Immunoglobulin A, Unpleasantness and ERP Activity

**DOI:** 10.1371/journal.pone.0030761

**Published:** 2012-02-02

**Authors:** Wencai Zhang, Fan Li, Shaozheng Qin, Jing Luo

**Affiliations:** 1 Key Laboratory of Mental Health, Institute of Psychology, Chinese Academy of Sciences, Beijing, China; 2 Department of Psychiatry and Behavioral Sciences, Stanford University School of Medicine, Stanford, California, United States of America; 3 Beijing Key Laboratory of Learning and Cognition, Department of Psychology, Capital Normal University, Beijing, China; University of Granada, Spain

## Abstract

Although the regulatory role of cognitive reappraisal in negative emotional responses is widely recognized, this reappraisal's effect on acute saliva secretory immunoglobulin A (SIgA), as well as the relationships among affective, immunological, and event-related potential (ERP) changes, remains unclear. In this study, we selected only people with low positive coping scores (PCSs) as measured by the Trait Coping Style Questionnaire to avoid confounding by intrinsic coping styles. First, we found that the acute stress of viewing unpleasant pictures consistently decreased SIgA concentration and secretion rate, increased perceptions of unpleasantness and amplitude of late positive potentials (LPPs) between 200–300 ms and 400–1000 ms. After participants used cognitive reappraisal, their SIgA concentration and secretion rate significantly increased and their unpleasantness and LPP amplitudes significantly decreased compared with a control condition. Second, we found a significantly positive correlation between the increases in SIgA and the decreases in unpleasantness and a significantly negative correlation between the increases in SIgA and the increases in LPP across the two groups. This study is the first to demonstrate that cognitive reappraisal reverses the decrease of SIgA. In addition, it revealed strong correlations among affective, SIgA and electrophysiological changes with convergent multilevel evidence.

## Introduction

Cognitive reappraisal refers to interpreting a situation's meaning in a way that alters its emotional impact. For instance, reappraising a stressor (e.g., a snake) can alter one's psychological and physiological responses (e.g., the snake is not harmful) [1], [2]. Although cognitive reappraisal is typically known as a down-regulation strategy to reduce the unpleasant emotional arousal evoked by a stressful event, this strategy also efficiently increases unpleasant emotions by re-interpreting a negative stimulus as even worse [3]–[5], or modifies a pleasant emotional stimulus as less pleasing [6]. Synthesizing evidence from affective, psychophysiological, and imaging studies suggests that cognitive reappraisal affects emotional and physiological arousal [1], [7] and produces changes in electrophysiological and hemodynamic activities during viewing affective pictures [5], [8]–[11]. For example, the cognitive reappraisal of a negative emotion decreased subjective unpleasantness and physiological arousal as measured by heart rate, galvanic skin response and blood pressure [1], [7]. Event-related potential (ERP) studies found that cognitive reappraisal with decreasing unpleasant or pleasant emotional responses both attenuated the amplitude of late positive potentials (LPPs) by approximately 400–1000 ms during affective picture viewing [6], [9], [10]. Later studies also found that cognitive reappraisals with increasing or decreasing negative emotions corresponded with enhancing or attenuating LPPs between approximately 200–300 ms and 400–1000 ms [3]–[5]. In addition, functional magnetic resonance imaging (fMRI) studies have suggested that a network consisting of the amygdala and the dorsal prefrontal cortex mediate these effects by regulating emotional processing and appraisal [12]. These studies convincingly indicate that the cognitive reappraisal strategy has a significant regulatory effect on negative emotional arousal using several methodologies.

However, how cognitive reappraisal alters immune responses, such as salivary immunity measured by secretory immunoglobulin A (SIgA), to negative emotion remains unclear. Given that there is considerable evidence linking psychological stress with immune dysregulation [13], it is conceivable to propose that psychological intervention, especially one that is targeted at stress reduction, will alleviate stress-related immune dysregulation. However, a meta-analytic review revealed weak and inconsistent evidence for this [14]. According to the model that posits that stress-management intervention alleviates immune dysregulation by modifying psychobiological processes set into motion by stressful experience, psychological stress could evoke negative emotional response, which could in turn induce immune dysregulation by activating fibers of the sympathetic division of the autonomic nervous system or by activating hormonal systems (including the hypothalamic-pituitary-adrenal axis, the sympathetic adrenal-medullary axis, and the hypothalamic pituitary-ovarian axis) [14], [15]. Stress management intervention, however, could possibly interrupt this dysregulating process by diminishing negative emotional responses. For example, cognitive restructuring through reinterpreting stressful circumstances as less threatening could diminish negative emotional responses that cause immune dysregulation [16], [17]. Further, it was suggested that stress-management intervention will be most successful at modulating immune responses when it fulfills three conditions: 1) the immune processes measured demonstrate sensitivity to stress and can hence be expected to change with successful intervention; 2) the intervention can successfully reduce stress; and 3) the stressful experience encountered by participants can impair immune function [14].

On the basis of these considerations, in this study, we managed to achieve these standards in three aspects: 1) We took SIgA, which was known to be important in preventing infection and to be sensitive to stressful experiences [14], [18], [19], as the index of immune responses. The two most commonly used measures of SIgA production in the field of psychoneuroimmunology have been SIgA concentration (the amount of total IgA protein present in a certain volume of saliva, i.e., µg/ml) and SIgA secretion rate (the amount of IgA protein detected per unit time, i.e., mg/minute). The two measures do not show completely consistent responses to stress, but they have the similar immunological meaning, i.e. the greater their value, the stronger the mucosal immune functioning [19]. 2) We took cognitive reappraisal as regulatory strategy. Cognitive reappraisal is well documented to be able to not only reduce stress experienced in viewing unpleasant pictures but also exert a highly specific and immediate regulation at almost the same time that a stressor (an unpleasant picture) is encountered. 3) We used negative affective pictures, which were selected from the standardized International Affective Picture System, as materials to induce stress. Such pictures are widely used in studies on emotion and negative emotion. In order to control for individual difference in intrinsic tendency to use cognitive reappraisal strategies [20], [21] and therefore successfully produce consistent inhibitory effects on SIgA immunity, we selected people with low positive coping scores (PCSs) as participants, who did not show a tendency to use cognitive reappraisal strategies when faced with stressful situations until the experimenter taught them to do so. This enables us to obtain a consistent inhibitory effect of negative emotional arousal on SIgA immunity and to further examine whether cognitive reappraisal regulation reverses this tendency. In sum, we have three predictions in this study: a) the SIgA immunity of the participants will show an acute decline after they have viewed the unpleasant pictures; b) applying cognitive reappraisal will reverse this tendency; and c) SIgA immunity improvement will be significantly correlated with other reappraisal-induced changes, such as decreased unpleasantness and LPPs.

Prediction a) was consistent with findings indicating the possibility that SIgA might rapidly decrease when pain is experienced (e.g., dental treatment or a cold pressor test) or unpleasant scenes are viewed [22]–[26]. Despite the fact that controversial evidence indicated that SIgA increased for some stressful tasks, such as mental arithmetic, memory tests, and exams [23], [27]–[30], meta-analyses suggested that the discrepancy in results regarding SIgA changes to stressful experiences might be caused by a lack of control of individual differences, especially stress-coping styles [31], [32]. In this study, we controlled for individual differences by selecting people with low PCSs as participants, and so we may have the opportunity to obtain consistently declined SIgA responses after stressful experiences.

Prediction b) was consistent with experimental observations that linked cognitive reappraisal with better immune function during stress: our previous study found that participants with higher PCSs and the intrinsic tendency to use cognitive reappraisal in processing unpleasant pictures demonstrated an immediate SIgA increase in stress [20]. Koh et al. found that the personality characteristic of positive reappraisal assessed by a questionnaire was linked with improved immune function [33]. Others have found that reappraisal-related characteristics, such as optimism and active coping, are correlated with better immune function during stress [34]–[36]. Accordingly, we may predict that, for the low PCS participants who have no intrinsic tendency to use cognitive reappraisal strategy, their immune responses would show dysregulation after stressful experiences, and this tendency would be significantly eliminated or even reversed by the application of cognitive reappraisal strategy.

Prediction c) is important for demonstrating the mechanism through which cognitive reappraisal alleviates stress-related immune dysregulation. That is, if increases in SIgA immunity were significantly correlated with other reappraisal-induced changes, such as decreased subjective unpleasantness and LPPs, then we can more convincingly infer that the reason that cognitive reappraisal removes stress-related immune dysregulation is related to the function of cognitive reappraisal in reducing one's negative emotional arousal during stress, as indexed by one's unpleasantness level and emotion-related LPPs. As stated by some investigators, multilevel models that link measures of behavioral, experiential, and physiological responses and their neural substrates provide a richer and deeper account of a phenomenon of interest than a single-level model by simultaneously drawing upon all levels of analysis [12], .

Thus, we used a two-group pretest-posttest paradigm [38] in which participants underwent a baseline day with no reappraisal and a test day with reappraisal after viewing highly negative emotionally arousing pictures on two separate days. This method allows us to obtain reliable baseline measurements, thereby avoiding potential baseline contamination caused by an alternating passive viewing/reappraisal condition within-group design. Based on the aforementioned considerations, the present study illustrates the acute protective effect of cognitive reappraisal on stress-related immunity and examines the relationship among the affective, immunological, and ERP changes.

## Methods

### Ethics statements

All participants were free of medication and provided written informed consent in accordance with the Declaration of Helsinki. The ethics committee of the Institute of Psychology, Chinese Academy of Sciences approved this study, its participant-recruitment procedure and its methodology.

### Participants

Thirty-two healthy undergraduates (mean age = 22.44±1.46 yrs) with normal or corrected-to-normal vision participated in this study. Participants were selected from a pool of 134 women based on their coping styles assessed by Trait Coping Style Questionnaire (TCSQ). Because several studies suggest that women have better memories for negative visual material compared with men [39], [40], only the former sex was included to avoid gender differences in response to negative imagery. A previous study suggested that participants whose SIgA increased after viewing unpleasant pictures had higher PCSs and more frequently applied cognitive reappraisal compared with those whose SIgA had decreased [20]; thus, we only included participants with low positive coping subscale scores (mean score = 28.66±3.36) who seldom used cognitive reappraisal strategies if not taught. Participants were randomly assigned to either the control group [mean age = 22.25±1.44; mean score = 29.06±2.57] or the reappraisal group [mean age = 22.63±1.50; mean score = 28.25±4.04]. There were no significant age [*t*(30) = 0.72, *P*>0.05] or score [*t*(30) = −0.68, *P*>0.05] differences.

### Stimuli

Two hundred negative non-face images [valence = 2.73±0.55; arousal = 5.80±0.74], chosen from the International Affective Picture System [41] and the Chinese Affective Picture System (CAPS) for the Chinese population [42] were used as stimuli in the affective challenge task to induce negative emotional arousal. These pictures (with a resolution of 72 pixels/inch and sized at 10 cm×7 cm) were divided into two equivalent sets by their valence and arousal. In addition, we ensured that an approximately equal number of images of bodily residual, snakes, soiled items, and so on were assigned to each set of pictures. One set of pictures were presented to half of the participants in each group for the baseline day, and the other were presented to them in the test day seven days later; this two sets of pictures in reverse order were presented to the other half of participants. Thus, the presentation order was counterbalanced across participants.

### Reappraisal training

We wanted to test whether applying cognitive reappraisal would influence affective, immunological, or electrophysiological responses caused by viewing unpleasant pictures. Therefore, a key manipulation of this study was to allow the participants in the reappraisal group to learn to use cognitive reappraisal while watching unpleasant IAPS and CAPS pictures. These participants were instructed to use a cognitive reappraisal strategy by generating an interpretation of or a story about each picture that explained the apparent negative events in a less negative way (e.g., women depicted crying outside a church could be described as attending a wedding rather than a funeral) [43]. Participants were trained intensively and completed 10 practice trials. At the end of the training, all participants reported that they were skilled in using these strategies to reinterpret unpleasant pictures. During the training period, the control group also completed 10 practice trials, but did not receive any coping strategy instructions.

### Overview of the procedure

The present study adopted a 2 (control and reappraisal groups)×2 (baseline and test days)×2 (pretest and posttest) factorial design. On the first day, baseline measurements for unpleasantness level, immune responses and ERP activities to the affective challenge task were obtained from both groups while participants passively viewed the pictures. Seven days later, participants returned to receive (the reappraisal group) or not receive (the control group) cognitive reappraisal strategy training. Afterward, all participants re-experienced an unpleasant picture presentation. During the training period, the control group did not receive any coping strategy instructions; these participants were simply asked to perform the same procedure as they did in the baseline day. The reappraisal group was instructed to use a cognitive reappraisal strategy when viewing unpleasant pictures. For the two groups, we collected ERP data during the task and collected the SIgA and unpleasant level of emotional states before (pretest) and after (posttest) the task (i.e., the affective challenge task) for both the initial baseline day and the final test day (see Figure 1). These pretest/posttest data allowed us to observe whether the affective challenge task reduced subjective unpleasantness and SIgA immunity, as well as whether cognitive reappraisal improves these elements.

**Figure 1:** Experimental procedure. (A) The general procedure consists of a baseline day (day 1) and a test day (7 days later). On the baseline day, the participants of the control and reappraisal groups were asked to passively view the pictures. On the test day, the participants of the control group were again asked to passively view the pictures; however, the participants of the reappraisal group were asked to generate positive reinterpretations for the presented pictures. Both on the baseline and the test day, ERP was collected during, and SIgA samples (T1 & T2) and unpleasantness level of emotional states (R1 & R2) were collected before and after, the unpleasant pictures presentation block. (B) Timeline for events during each trial. Each picture was presented for 6 s with a random inter-stimulus interval of 0.8–1.2 s, during which a fixation cross was presented.

#### Baseline day (Day 1)

We obtained the baseline measurements on the first day including unpleasantness level, SIgA and ERP using identical procedures for both the control and reappraisal groups. Upon arriving at the laboratory, all participants gargled and rinse their mouths and then rest for 10 minutes in a soundproof room. A pretest saliva sample (T1) was collected from participants during this rest state. At the same time, participants reported their current feelings of unpleasantness on a nine-point scale from 1 (unpleasant) to 9 (pleasant). The participants then viewed unpleasant pictures. After a brief practice session, participants passively viewed 100 negative emotionally arousing pictures while their synchronous EEG activity was recorded in a formal experimental block. Each picture was presented for 6 s interleaved with a random inter-stimulus interval that varied from 0.8 s to 1.2 s during which a black screen with a fixation cross was presented. Participants passively viewed the unpleasant pictures and to pressed the spacebar when the picture disappeared from the screen. The participants were instructed to make a simple dichotomous judgment (e.g., either “I feel unpleasant” or “I feel very unpleasant”) immediately after each picture presentation to ensure the participants were engaged in attentively perceiving the pictures. After the formal experimental condition, a posttest saliva sample (T2) was collected, and participants were again asked to reported their current emotional state of unpleasantness on a nine-point scale again. The pretest and posttest differences in the SIgA and unpleasant ratings indicated changes induced by the stimuli.

#### Test day (7 days later)

Seven days after the baseline assessments, procedures similar to those during the first day were applied. This time, however, before participants viewed another set of 100 unpleasant pictures, those in the reappraisal group received cognitive reappraisal coping strategy guidance, whereas participants in the control group simply repeated the same procedure as on Day 1. The participants then completed a formal experimental block and reappraised each picture. Finally, to determine whether the participants reappraised the pictures during the formal experimental block, we randomly selected 10 pictures from the experimental block and presented them to the participants. Participants recalled and orally reported their cognitive reappraisal strategies while viewing the target pictures, and their responses were recorded to examine how they applied the cognitive reappraisal strategy. Two psychology experts, who were blinded to the present study, judged these reports. These experts received training in CBT and were quite experienced in judging the cognitive reappraisal strategies used in the processing of affective pictures. They provided a “yes” or “no” response to assess whether participants “applied a reappraisal strategy” for each picture. The reappraisal scores for each participant were computed by counting the number of “yes” responses. Finally, a Pearson's correlation was computed between the two experts to check the consistency of their judgments. The procedure used to collect saliva samples, EEG data and unpleasantness level were the same as on the first day.

### Saliva collection and SIgA measurement

Saliva samples were collected at pretest and posttest at the baseline and test day. Thus, each participant had four saliva samples taken (see Figure 1). Participants were asked to gargle and rinse their mouths. An aseptic cotton swab was then placed underneath their tongues for 2 minutes during which time they avoided swallowing and chewing. Thus, saliva accumulated on the floor of their mouths absent of salivary secretion stimulation by any means of oro-facial movements. Saliva was first separated from the cotton swab by centrifugation at 4800 rpm for 5 minutes and then placed in a centrifuge tube sealed and frozen at −20°C for later analysis. The amount of saliva in grams was converted to milliliters assuming a saliva density of 1 g/ml. We measured salivary SIgA concentrations using an enzyme-linked immunosorbent assay (ELISA). SIgA secretion rate (µg/minute) was calculated by multiplying the absolute SIgA concentration (µg/ml) by the saliva flow rate (ml/minute), the latter of which was calculated by dividing the total volume of saliva obtained in each sample (ml) by the time taken to produce the sample (minute) [44]. One control group participant was excluded from further analyses because his SIgA concentration was undetectable (i.e., it was under the minimum detection threshold of the standard substance of ELISA).

### ERPs

While participants viewed unpleasant pictures, (EEG was recorded from 64 scalp sites using Ag/AgCl electrodes mounted within an elastic cap (Neuroscan Inc.). The reference was the computed value of average mastoids. When the EEG was recording, all of the scalp sites and the right mastoid were referenced to the left mastoid. The average mastoids reference derivation for a given site was computed off-line using the formula a′ = a−(r/2), where a′ is the desired value for a site with averaged mastoids reference, and a and r are the recorded values of this site and the right mastoid, respectively. The vertical and horizontal electrooculograms (VEOG and HEOG, respectively) were recorded using two pairs of electrodes; one pair was placed above and below the left eye, and another pair was placed 10 mm from the outer canthi of both eyes. In data acquisition online all interelectrode impedances were maintained at 0.5 kΩ. A bandpass of 0.05–100 Hz was used for the recording amplifiers and digitized at 500 Hz in the EEG data acquisition online. Then in data processing offline EEG data were digitally filtered using a 30 Hz low-pass and were epoched into 1800-ms periods (including a 300-ms pre-stimulus baseline). Ocular artifacts were removed from the EEG signal using a regression procedure implemented in the Neuroscan software [45]. Trials with various artifacts were rejected using a criterion of ±75 mV. We analyzed the following 15 sites: F3, F4, Fz, FC3, FC4, FCz, C3, C4, Cz, CP3, CP4, CPz, P3, P4, and Pz. The mean amplitudes were measured in the early LPP of 200–300 ms and the late LPP of 400–1000 ms. We analyze the ERP data in the 200–300 ms and 400–1000 ms ranges for two reasons. First, Olofsson et al. reviewed ERP findings on affective picture processing in recent years and focused primarily on the two latencies at the earlier component (200–300 ms) and the later component (>300 ms) [46]. Second, previous studies of cognitive reappraisal found the activities at the earlier component (200–300 ms) and LPP (most limited in the 300–1000 ms range) differed between the regulation and control conditions and suggested that LPP modulation by cognitive reappraisal began just 200 ms after the onset of emotional stimuli [3], [4]. Hajcak and Nieuwenhuis (2006) specifically called these LPP [9]. In the present study, the components of 200–300 ms and 400–1000 ms are known as early LPP and late LPP.

### Data analyses

Because this study collected complicated multilevel data, we describe the specific data analyses for this dataset.

First, the unpleasantness level, SIgA concentrations and secretion rate were separately collected four times at pretest and posttest at the baseline and test days. Pretest differences between groups might systematically bias the interpretations of posttest differences [38]; thus, we conducted an independent t-test for each measure separately to examine whether the between-group pretests at the baseline and test days were equal. If the between-group pretest for a given measure was equal (i.e., no significant difference), then we conducted a 2×2×2 repeated-measures analyses of variance (ANOVA) to examine the main and interaction effects within test (i.e., pretest and posttest), day (i.e., baseline and test) and group (i.e., control and reappraisal). If the interaction effect was significant, then we conducted simple effect analyses using t-tests; however, if the between-group pretest for a given measure was unequal (i.e., significantly different), then a separate analysis of covariance (ANCOVA) analyzed the between-group effect within the baseline and test days. This analytic plan is the preferred method to examine data obtained from a pretest/posttest paradigm to eliminate systematic bias [38].

Second, ERP data were collected at the baseline and test days. Similar to examining the equality of the pretest unpleasantness level and SIgA immunities between groups, we first examined whether the baseline ERPs were equal with regard to the early and late LPP components between the reappraisal and control groups. We conducted this test using an ANOVA instead of an independent t-test because 15 representative electrode sites were considered. If the baseline ERPs were unequal between groups, then an ANOVA (not an ANCOVA) was applied to the change scores that were computed by subtracting the baseline recordings from the reappraisal recordings at each electrode site, to analyze the early and late LPP components among the control and reappraisal groups. In this case, ANCOVA is not suitable for ERP data because it would use the 15 electrodes sites as potential covariates, which might lead to results that are difficult to explain. Applying the change scores of the test day minus the baseline day is an alternative method of analyzing data obtained from a pretest/posttest paradigm to eliminate systematic bias [38]. In addition, we compared test-day with baseline-day ERPs using ANOVAs for the control and reappraisal groups to observe the differences for each group.

Third, we conducted Pearson's correlation analyses on unpleasantness level, SIgA concentrations, secretion rates and ERPs using the two groups' change scores. The change scores of the unpleasantness level, SigA concentration and secretion rate were computed by the measure of test day (posttest minus pretest) minus the measure of baseline day (posttest minus pretest). The LPP change scores were computed by averaging change scores of the measure of test day minus the measure of baseline day across the 15 electrode sites.

## Results

### Expert judgments

There was a significant correlation between the two judges [*r* = 0.969, *P*<0.001], indicating high consistency in their judgments. The average reappraisal rate for the 10 selected pictures was 0.988, which indicates that nearly every participant in the reappraisal group applied cognitive reappraisal strategies for each picture.

### Self-reported affect

Independent t-tests did not show a significant difference in the pretest unpleasantness level in the baseline [*t*(29) = 1.81, *p*>0.05] and test days [*t*(29) = −0.035, *p*>0.05] with regard to the reappraisal and control groups, indicating that the between-group pretests are equal. Next ANOVA analysis revealed a significant three-way interaction [*F*(1, 29) = 18.06, *p*<0.001] among test (pretest and posttest), day (baseline and test) and group (control and reappraisal). As shown in Figure 2. For the baseline day, separate paired t-tests found significantly increased unpleasantness in the posttest compared with the pretest for both the control [*t*(14) = 5.17, *p*<0.001] and reappraisal groups [*t*(15) = 6.47, *p*<0.001]. For the test day, separate paired t-tests found significantly increased unpleasantness in the posttest compared with the pretest in the control group [*t*(14) = 5.34, *p*<0.001]. However, these findings did not hold for the reappraisal group [*t*(15) = 1.59, *p*>0.05]. These results indicate that passively viewing unpleasant pictures significantly increased control-group participants' perceptions of unpleasantness in both the baseline and test days. In contrast, passively viewing unpleasant pictures also significantly increased reappraisal-group participants' perceptions of unpleasantness in the baseline day but reappraising the unpleasant pictures prevented this increase of unpleasantness in the test day. An additional independent t-test revealed that the posttest unpleasantness of the reappraisal group in the test day were significantly larger than those of the control group [*t*(29) = 4.80, *p*<0.001]. This finding indicates that cognitive reappraisal significantly decreased subjective unpleasantness.

**Figure 2:** Changes of unpleasantness level. Unleasantness level at the pretest and posttest in the baseline and test days for the control and the reappraisal group. Notably, passively viewing unpleasant pictures significantly increased unpleasant (or decreased pleasantness) for both the two group. The unpleasantness significantly decreased in the reappraisal group in comparison to that of the control group.

### The effects of cognitive reappraisal on SIgA

Independent t-tests revealed significant pretest differences of SIgA concentration [*t*(29) = −2.65, *p*<0.05] and SIgA secretion rate [*t*(29) = −2.07, *p*<0.05] between the reappraisal and control groups during the baseline day. Similar tests revealed significant pretest differences of SIgA concentration [*t*(29) = −4.00, *p*<0.01] and SIgA secretion rate [*t*(29) = −2.74, *p*<0.05] between the reappraisal and control groups during the test day, indicating that the between-group pretests are different. Then using their corresponding pretest data in the test day as a covariate to conducted an ANCOVA, we found significantly increased posttest SIgA concentration [*F*(1, 28) = 11.19, *p*<0.01] and SIgA secretion rate [*F*(1, 28) = 11.03, *p*<0.01] in the reappraisal group compared with the control group (Figure 3, left and right). However, there were no significant differences observed for SIgA concentration and secretion rate [both *F*<1.0] in the baseline days between the control and reappraisal groups. These results indicate that the application of cognitive reappraisal in the reappraisal group significantly potentiated participant SIgA immune function compared with the control group. Paired t-tests for the baseline day revealed significantly decreased SIgA concentrations and secretion rates in the posttest than the pretest for both the control [concentration: *t*(14) = 4.50, *p*<0.01; secretion rate: *t*(14) = 5.23, *p*<0.01] and reappraisal groups [concentration: *t*(15) = 3.23, *p*<0.05; secretion rate: *t*(15) = 3.82, *p*<0.05]. For the test day, we also found a significantly decreased SIgA concentration [*t*(14) = 4.59, *p*<0.01] and secretion rate [*t*(14) = 4.84, *p*<0.01] in the posttest relative to the pretest for the control group. Conversely, we observed significantly increased SIgA concentrations [*t*(15) = −3.67, *p*<0.05] during the posttest compared with the pretest in the reappraisal group. These results indicate that passively viewing unpleasant pictures decreased the SIgA immune function at baseline for both groups. However, cognitive reappraisal potentiated SIgA immune function in the test day of the reappraisal group.

**Figure 3:** Changes of SIgA concentrations and SIgA secretion rates. SIgA concentrations (left) and SIgA secretion rates (right) in the pretest and posttest during the baseline and test days for the control and reappraisal group. Notably, both were significantly increased after cognitive reappraisal in the reappraisal group as compared to the control group.

### The effects of cognitive reappraisal on ERPs

As shown in Figure 4, we found significant changes in the mean amplitude of early LPP (200–300 ms) and late LPP (400–1000 ms) during the baseline and test days for the control and reappraisal groups. Firstly, we found a significant between-group main effect of the early LPPs (200–300 ms) [*F*(1, 29) = 6.57, *p*<0.05] in the baseline ERPs using an ANOVA, which indicates the baseline-day ERPs is unequal. Then an ANOVA with change scores found that there were significant between-group main effects in both early LPPs (200–300 ms) [*F*(1, 29) = 9.59, *p*<0.01] and late LPPs (400–1000 ms) [*F*(1, 29) = 8.03, *p*<0.01] (Figure 4, right). We also found significant interaction effect of group×electrode sites in the change scores of early LPP (200–300 ms) [*F*(1, 29) = 3.02, *p*<0.001]. Further independent t-test showed that reappraisal group showed most significant decrease of early LPP (200–300 ms) in the anterior electrode sites (including F3, F4, Fz, FC3, FC4, FCz, C3, C4, Cz, CP3, Pz, at least *p*<0.05) in comparison to control group. But we didn't found such an interaction effect for late LPP (400–1000 ms) [*F*(1, 29) = 1.25, *p*>0.05]. Furthermore, when contrasting the baseline day with the test day, there were significant decreases in early LPPs (200–300 ms) [*F*(1, 15) = 17.90, *p*<0.001] and late LPPs (400–1000 ms) [*F*(1, 15) = 7.08, *p*<0.05] (Figure 4, middle) for the reappraisal group but not for the control group (Figure 4, left). We also found significant interaction effect of day×electrode sites in the change scores of early LPP (200–300 ms) [*F*(1, 15) = 3.79, *p*<0.001] in the reappraisal group. Further paired t-test showed that reappraisal participants in the test day showed most significant decrease of early LPP (200–300 ms) in the anterior electrode sites (including F3, F4, Fz, FC3, FC4, FCz, C3, C4, Cz, CP3, CP4, Pz, at least *p*<0.05) in comparison to the baseline day. But we didn't found such an interaction effect for late LPP (400–1000 ms) [*F*(1, 15) = 3.791.73, *p*>0.05]. These results indicated that, reappraisal use of the reappraisal group in the test day could induce reliable decreases in both of early LPP (200–300 ms) and late LPP (400–1000 ms), whether compared with passive viewing of the control group who never learned how to use the strategies, or compared with passive viewing of the same reappraisal group in the baseline day, Moreover, the early LPP (200–300 ms) located in the anterior electrode sites exhibited reappraisal-induced significant decrease during viewing unpleasant pictures both when comparing reappraisal group with control group and when comparing reappraisal session with baseline session in the same reappraisal group. This implied the regulatory effects of cognitive reappraisal on negative arousal may be related to early attention function of frontal cortex.

**Figure 4:** Changes of LPP for the control and the reappraisal groups. Left column: Grand averages for the control group; Middle column: Grand averages for the reappraisal group. Right column: Difference waveforms between the baseline and test days for the control and reappraise groups.

### Relationships among the changes in affect, SIgA immune responses and ERPs

To further investigate the relationships among affective, immunological and ERP changes, correlation analyses of change scores in unpleasantness level, SIgA levels, and ERPs were conducted across the two groups (see the illustration in Data Analyses). The results indicated that: (1) an increased SIgA concentration is significantly negatively correlated with the increases in early LPP (200–300 ms) and late LPP (400–1000 ms) and is significantly positively correlated with decreased unpleasantness. (2) an increased SIgA secretion rate is significantly negatively correlated with increases in early LPP (200–300 ms) and late LPP (400–1000 ms). (3) an increased early LPP (200–300 ms) is significantly negatively correlated with decreased unpleasantness (Table 1). These results indicate that there is a general correlation among increased SIgA immunity, decreased unpleasantness, and early and late LPP changes. Figure 5 shows the correlation between the SIgA secretion rates and LPPs (400–1000 ms) (left) as well as between the SIgA concentrations and unpleasantness level (right).

**Figure 5:** The correlation among the SIgA, LPP, and unpleasantness level. Increased SIgA secretion rates is negatively correlated with increased LPP (left); and increased of SIgA concentrations is positively with decreased unpleasantness (or increased pleasantness) (right).

**Table 1:** Correlations among the changes in SIgA, ERPs and emotional states.

	Increased Early LPP(200–300 ms)	Increased Late LPP(400–100 ms)	Increased SIgA concentration (µg/min)	Increased SIgA secretion rate (µg/min)
Increased SIgA concentration (µg/min)	−0.43*	−0.41*	–	–
Increased SIgA secretion rate (µg/min)	−0.43*	−0.72***	–	–
Decreased unpleasantness	−0.37*	−0.22	0.52**	0.34

Note:

***p<0.001;

**p<0.01;

*p<0.05.

## Discussion

The present study investigated reappraisal-induced changes in negative affect, ERP and SIgA immunity. We found that cognitive reappraisal not only significantly reduced negative emotional arousal and the associated LPP amplitudes during stressful experiences, but also alleviated stress-induced SIgA dysregulation. In addition, we found significant correlations among in enhanced immune function, attenuated unpleasantness level and attenuated LPPs that further confirmed the relationships among these variables. This verifies the model suggesting cognitive reappraisal improves stress-induced SIgA dysregulation through a “psychological” pathway of reducing one's negative emotional arousal in stress [14].

### Cognitive reappraisal reversed the attenuated SIgA immunological response induced by negative emotion

As the most abundant immunoglobulin, mucosal SIgA constitutes the first line of defense of infection and disease prevention by interfering with microbial entry and multiplication [18]. The present study demonstrated that passively viewing unpleasant pictures significantly reduced low PCSs' SIgA concentrations, SIgA secretion rates and increased unpleasantness level in the baseline day of both the control and reappraisal groups without explicitly introducing any coping strategies. These results were consistent with previous findings showing that specific emotionally charged states (e.g., pain and disgust) weaken salivary SIgA immunity [22]–[26]. The decreased SIgA concentrations and secretion rates induced by acute stress probably reflect decreases in basolateral IgA availability [18]. These results indicate that acute emotional stress induces an attenuated SIgA immune function. Note that we kept the coping styles consistent across all participants by sampling those with low PCSs. This might help to obtain highly consistent SIgA attenuation patterns across participants (i.e., all participants showed reduced SIgA concentrations, and 87% of the sample indicated reduced SIgA secretion rates at baseline).

This study also demonstrated that cognitive reappraisal significantly reverses increased unpleasantness as well as decreased SIgA concentrations and secretion rates in the reappraisal group during the test day compared with the control group. These results illustrate that cognitive reappraisal is a valid strategy to decrease subjective unpleasantness and increase SIgA immune function. The SIgA-increased finding is generally in line with previous studies that have applied relaxation exercise, social support, and emotional expression [14], [47], [48], [49]–[52]; however, the present study has advantages over these studies. First, viewing the standard unpleasant pictures from IAPS produced an intensity-controlled stressful setting by balancing the valence in all conditions. Second, cognitive reappraisal exerts a real-time modulatory influence aimed at each stressful event (i.e., picture) and improves the concurrent negative emotional experience, whereas relaxation exercises and social support cannot administer this type of specific influence. Third, using a two-group pretest/posttest paradigm, we determined that cognitive reappraisal (and not repeated passive viewing) reversed the SIgA immunity effect because the SIgA immunity in the control group continued to decrease in the second viewing.

### The effects of cognitive reappraisal on the early and late LPP components

ERPs were recorded in addition to SIgA immunity data. Reappraising unpleasant stimuli significantly reduced early LPPs (200–300 ms) and late LPPs (400–1000 ms) compared with passive viewing. An analysis of the differences among waves suggested that the reappraisal group had greater decreases in early LPPs (200–300 ms) and late LPPs (400–1000 ms) compared with the control group. Moreover, the reappraisal-induced decrease in unpleasantness was negatively correlated with an increase in early LPPs (200–300 ms). Previous ERP studies found that cognitive reappraisals of unpleasant stimuli are associated with diminished LPPs compared with passive viewing conditions [3], [4], [9], [10], which indicates that LPPs are susceptible to top-down processing influences. LPPs are also highly sensitive to the emotional intensity of stimuli and exhibit higher magnitudes for both pleasant and unpleasant stimuli compared with neutral stimuli [53]–[55]. The present study observed similar LPP changes, which confirms that LPPs are sensitive to cognitive reappraisal and may be a useful indicator to detect the mechanisms responsible for successful emotion regulation.

### The relationships among negative affect, SIgA immunity and ERPs

Considering that cognitive reappraisal during emotion processing has a multilevel effect on affective, immunological, and neural activities, we examined the relationships among their changes scores across the two groups. We observed significant correlations among these variables. Specifically, increased SIgA concentrations, SIgA secretion rates and decreased unpleasantness were each negatively correlated with both early LPP (200–300 ms) and late LPP (400–1000 ms) increases. Moreover, increased SIgA concentrations was positively correlated with decreased unpleasantness. More specifically, it is posited that the early LPPs (200–300 ms) reflect early attentive allocation of emotion processing, whereas the late LPPs (400–800 ms) are associated with later emotional appraisals and arousal [56], [46]. And Gross and colleagues' model of Emotion Generation and Regulation proposed that emotion regulatory strategies may have an impact at any point in the emotion-generative process including the situation, attention, appraisal and/or response stages, in sequence [2], [ 57]. Therefore, these correlative evidences obtained from multilevel data are helpful in illustrating the inhibitory regulation effect of cognitive reappraisal played on the early attention (e.g., early LPP decrease) and late appraisal stages in the processing of negative emotion (e.g., late LPP decrease) are both related to decreased unpleasantness and increased immune responses. Thus, this study not only provides direct evidence for the statement that cognitive reappraisal is a system of adaptive control that may be observed at the level of physiological, attentional, emotional, behavioral, cognitive, and interpersonal/social processes [37], but also supports the theoretical framework that proposed a) cognitive reappraisal, as one of the key components of stress-management intervention, could remove (or even reverse) the stress-related immune dysregulation; and b) cognitive reappraisal makes this achievement through regulating the negative emotion evoked in stressful experience [14]

Although this study firmly demonstrates that cognitive reappraisal reverses the attenuation of SIgA immunity and indicates that reappraisal-induced LPP changes are associated with improved SIgA immunity and emotional experience, it also has some limitations. First, its sample size (16 females in each group) was relatively small; additional experiments with larger sample sizes might be more informative and more representative of the population. Second, although we attempted to ensure that there would be differences between receiving and not receiving reappraisal training by selecting the participants with low PCS who were considered to have almost no intrinsic reappraisal tendencies and by consistent judgements made by the two experts that almost all participants in the former group had applied cognitive reappraisal strategies. However, these jobs could not completely confirm that the reappraisal group actually applied the cognitive reappraisal strategy relative to the control group because these experts only made judgments on the reappraisal group. This methodology could be improved in future research if these judgments were performed for both groups.

## References

[1] Gross JJ, John OP (2003). Individual differences in two emotion regulation processes: implications for affect, relationships, and well-being.. Journal of Personality and Social Psychology.

[2] Gross JJ, Thompson RA, Gross JJ (2007). Emotion regulation: conceptual foundation.. Handbook of emotion regulation.

[3] Moser JS, Hajcak G, Bukay E, Simons RF (2006). Intentional modulation of emotional responding to unpleasant pictures: an ERP study.. Psychophysiology.

[4] Moser JS, Krompinger JW, Dietz J, Simons RF (2009). Electrophysiological correlates of decreasing and increasing emotional responses to unpleasant pictures.. Psychophysiology.

[5] Moser JS, Most SB, Simons RF (2010). Increasing negative emotions by reappraisal enhances subsequent cognitive control: a combined behavioral and electrophysiological study.. Cognitive, Affective & Behavioral Neuroscience.

[6] Krompinger JW, Moser JS, Simons RF (2008). Modulations of the electrophysiological response to pleasant stimuli by cognitive reappraisal.. Emotion.

[7] Gross JJ (2002). Emotion regulation: affective, cognitive, and social consequences.. Psychophysiology.

[8] Ochsner KN, Ray RD, Cooper JC, Robertson ER, Chopra S (2004). For better or for worse: neural systems supporting the cognitive down- and up-regulation of negative emotion.. Neuroimage.

[9] Hajcak G, Nieuwenhuis S (2006). Reappraisal modulates the electrocortical response to unpleasant pictures.. Cognitive, Affective & Behavioral Neuroscience.

[10] Foti D, Hajcak G (2008). Deconstructing reappraisal: descriptions preceding arousing pictures modulate the subsequent neural response.. Journal of Cognitive Neuroscience.

[11] McRae K, Hughes B, Chopra S, Gabrieli JD, Gross JJ (2010). The Neural Bases of Distraction and Reappraisal.. Journal of Cognitive Neuroscience.

[12] Ochsner KN, Gross JJ (2008). Cognitive emotion regulation: insights from social cognitive and affective neuroscience.. Current Directions in Psychological Science.

[13] Herbert TB, Cohen S (1993). Stress and immunity in humans: A meta-analytic review.. Psychosomatic Medicine.

[14] Miller GE, Cohen S (2001). Psychological interventions and the immune system: a meta-analytic review and critique.. Health Psychology.

[15] Blalock JE (1994). The syntax of neuroendocrine-immune communication.. Immunology Today.

[16] Antoni MH, Baggett L, Ironson G, LaPerriere A, August S (1991). Cognitivebehavioral stress management intervention buffers distress responses and immunologic changes following notification of HIV-1 seropositivity.. Journal of Consulting and Clinical Psychology.

[17] Lutgendorf SK, Antoni MH, Ironson G, Klimas NG, Kumar M (1997). Cognitive-behavioral stress management decreases dysphoric mood and herpes simplex virus-type 2 antibody litres in symptomatic HIV-seropositive gay men.. Journal of Consulting and Clinical Psychology.

[18] Bosch JA, Ring C, de Geus EJ, Veerman EC, Amerongen AV (2002). Stress and secretory immunity.. International Review of Neurobiology.

[19] Valdimarsdottir HB, Stone AA (1997). Psychosocial factors and secretory immunoglobulin A.. Critical Reviews in Oral Biology and Medicine.

[20] Li F, Han BX, Ren J, Luo J (2008). Effects of negative emotion and its correlated neural activity on secretory immunoglobulin A.. Chinese Science Bulletin.

[21] Drabant EM, McRae K, Manuck SB, Hariri AR, Gross JJ (2009). Individual differences in typical reappraisal use predict amygdala and prefrontal responses.. Biological Psychiatry.

[22] Willemsen G, Carroll D, Ring C, Drayson M (2002). Cellular and mucosal immune reactions to mental and cold stress: associations with gender and cardiovascular reactivity.. Psychophysiology.

[23] Ring C, Harrison LK, Winzer A, Carroll D, Drayson M (2000). Secretory immunoglobulin A and cardiovascular reactions to mental arithmetic, cold pressor, and exercise: effects of alpha-adrenergic blockade.. Psychophysiology.

[24] Kugler J, Breitfeld I, Tewes U, Schedlowski M (1996). Excavation of caries lesions induces transient decrease of total salivary immunoglobulin A concentration.. European Journal of Oral Sciences.

[25] Hennig J, Pössel P, Netter P (1996). Sensitivity to disgust as an indicator of neuroticism: A psychobiological approach.. Personality and Individual Differences.

[26] Bosch JA, de Geus EJ, Kelder A, Veerman EC, Hoogstraten J (2001). Differential effects of active versus passive coping on secretory immunity.. Psychophysiology.

[27] Carroll D, Ring C, Shrimpton J, Evans P, Willemsen G (1996). Secretory immunoglobulin A and cardiovascular responses to acute psychological challenge.. International Journal of Behavioral Medicine.

[28] Ring C, Carroll D, Willemsen G, Cooke J, Ferraro A (1999). Secretory immunoglobulin A and cardiovascular activity during mental arithmetic and paced breathing.. Psychophysiology.

[29] Winzer A, Ring C, Carroll D, Willemsen G, Drayson M (1999). Secretory immunoglobulin A and cardiovascular reactions to mental arithmetic, cold pressor, and exercise: effects of beta-adrenergic blockade.. Psychophysiology.

[30] Willemsen G, Ring C, McKeever S, Carroll D (2000). Secretory immunoglobulin A and cardiovascular activity during mental arithmetic: effects of task difficulty and task order.. Biological Psychology.

[31] Denson TF, Spanovic M, Miller N (2009). Cognitive appraisals and emotions predict cortisol and immune responses: a meta-analysis of acute laboratory social stressors and emotion inductions.. Psychological Bulletin.

[32] Segerstrom SC, Miller GE (2004). Psychological stress and the human immune system: a meta-analytic study of 30 years of inquiry.. Psychological Bulletin.

[33] Koh KB, Lee Y, Beyn KM, Chu SH, Kim DM (2008). Counter-stress effects of relaxation on proinflammatory and anti-inflammatory cytokines.. Brain, Behavior, and Immunity.

[34] Segerstrom SC, Taylor SE, Kemeny ME, Fahey JL (1998). Optimism is associated with mood, coping, and immune change in response to stress.. Journal of Personality and Social Psychology.

[35] Koolhaas JM (2008). Coping style and immunity in animals: making sense of individual variation.. Brain, Behavior, and Immunity.

[36] Zozulya AA, Gabaeva MV, Sokolov OY, Surkina ID, Kost NV (2008). Personality, coping style, and constitutional neuroimmunology.. Journal of Immunotoxicology.

[37] Calkins SD (2009). Commentary: Conceptual and Methodological Challengesto the Study of Emotion Regulation and Psychopathology.. Journal of Psychopathology and Behavioral Assessment.

[38] Dimitrov DM, Rumrill PD (2003). Pretest-posttest designs and measurement of change.. Work.

[39] Cahill L, Haier RJ, White NS, Fallon J, Kilpatrick L (2001). Sex-related difference in amygdala activity during emotionally influenced memory storage.. Neurobiology of Learning and Memory.

[40] Canli T, Desmond JE, Zhao Z, Gabrieli JD (2002). Sex differences in the neural basis of emotional memories.. Proceedings of the National Academy of Sciences of the United States of America.

[41] Lang PJ, Bradley MM, Cuthbert B (2001).

[42] Bai L, Ma H, Huang YX, Luo YJ (2005). The Development of Native Chinese Affective Picture System-A pretest in 46 College Students.. Chinese Mental Health Journal.

[43] Ochsner KN, Bunge SA, Gross JJ, Gabrieli JD (2002). Rethinking feelings: an FMRI study of the cognitive regulation of emotion.. Journal of Cogntive Neuroscience.

[44] Matsubara Y, Shimizu K, Tanimura Y, Miyamoto T, Akimoto T (2010). Effect of acupuncture on salivary immunoglobulin A after a bout of intense exercise.. Acupuncture Medicine.

[45] Semlitsch HV, Anderer P, Schuster P, Presslich O (1986). A solution for reliable and valid reduction of ocular artifacts, applied to the P300 ERP.. Psychophysiology.

[46] Olofsson JK, Nordin S, Sequeira H, Polich J (2008). Affective picture processing: an integrative review of ERP findings.. Biological Psychology.

[47] Taniguchi T, Hirokawa K, Tsuchiya M, Kawakami N (2007). The immediate effects of 10-minute relaxation training on salivary immunoglobulin A (s-IgA) and mood state for Japanese female medical co-workers.. Acta Medicinae Okayama.

[48] Pawlow LA, Jones GE (2005). The impact of abbreviated progressive muscle relaxation on salivary cortisol and salivary immunoglobulin A (sIgA).. Applied Psychophysiology and Biofeedback.

[49] Ohira H (2004). Social support and salivary secretory immunoglobulin A response in women to stress of making a public speech.. Perceptual and Motor Skills.

[50] Takagi S, Ohira H (2004). Effects of expression and inhibition of negative emotions on health, mood states, and salivary secretory immunoglobulin A in Japanese mildly depressed undergraduates.. Perceptual and Motor Skills.

[51] Barling NR, Raine SJ (2005). Some effects of hypnosis on negative affect and immune system response.. Australian Journal of Clinical & Experimental Hypnosis.

[52] Reid MR, Mackinnon LT, Drummond PD (2001). The effects of stress management on symptoms of upper respiratory tract infection, secretory immunoglobulin A, and mood in young adults.. Journal of Psychosomatic Research.

[53] Cuthbert BN, Schupp HT, Bradley MM, Birbaumer N, Lang PJ (2000). Brain potentials in affective picture processing: covariation with autonomic arousal and affective report.. Biological Psychology.

[54] Schupp HT, Cuthbert BN, Bradley MM, Cacioppo JT, Ito T (2000). Affective picture processing: the late positive potential is modulated by motivational relevance.. Psychophysiology.

[55] Schupp HT, Junghofer M, Weike AI, Hamm AO (2004). The selective processing of briefly presented affective pictures: an ERP analysis.. Psychophysiology.

[56] Dien J, Spencer KM, Donchin E (2004). Parsing the late positive complex: mental chronometry and the ERP components that inhabit the neighborhood of the P300.. Psychophysiology.

[57] Gross JJ (1998). Antecedent- and response-focused emotion regulation: divergent consequences for experience, expression, and physiology.. Journal of Personality and Social Psychology.

